The article "Fully Convolutional Network and Visual Saliency-Based Automatic Optic Disc Detection in Retinal Fundus Images" was published in 2021. Journal: J Healthc Eng.

# Fully Convolutional Network and Visual Saliency-Based Automatic Optic Disc Detection in Retinal Fundus Images

**DOI:** 10.1155/2021/3561134

**Published:** 2021-08-31

**Authors:** Xiaosheng Yu, Ying Wang, Siqi Wang, Nan Hu

**Affiliations:** ^1^Faculty of Robot Science and Engineering, Northeastern University, Shenyang 110819, China; ^2^College of Information Science and Engineering, Northeastern University, Shenyang 110819, China; ^3^School of Information and Control Engineering, Shenyang Jianzhu University, Shenyang 110168, China

## Abstract

We present in this paper a novel optic disc detection method based on a fully convolutional network and visual saliency in retinal fundus images. Firstly, we employ the morphological reconstruction-based object detection method to locate the optic disc region roughly. According to the location result, a 400 × 400 image patch that covers the whole optic disc is obtained by cropping the original retinal fundus image. Secondly, the Simple Linear Iterative Cluster approach is utilized to segment such an image patch into many smaller superpixels. Thirdly, each superpixel is assigned a uniform initial saliency value according to the background prior information based on the assumption that the superpixels located on the boundary of the image belong to the background. Meanwhile, we use a pretrained fully convolutional network to extract the deep features from different layers of the network and design the strategy to represent each superpixel by the deep features. Finally, both the background prior information and the deep features are integrated into the single-layer cellular automata framework to gain the accurate optic disc detection result. We utilize the DRISHTI-GS dataset and RIM-ONE r3 dataset to evaluate the performance of our method. The experimental results demonstrate that the proposed method can overcome the influence of intensity inhomogeneity, weak contrast, and the complex surroundings of the optic disc effectively and has superior performance in terms of accuracy and robustness.

## 1. Introduction

Glaucoma is one of the most common ocular diseases which can cause loss of vision and blindness. By 2020, about 80 million people worldwide suffer from this disease. Glaucoma is a disease characterized by atrophy of the optic nerve head (ONH), the progressive of retinal ganglion cells, and decreased vision [1]. The main factors leading to glaucoma are the increased intraocular pressure and the insufficient blood supply to the optic nerve in the optic disc. The other factors include family history, genetics, race, and age. The loss of vision caused by glaucoma is totally irreversible and extremely harmful. Therefore, early diagnosis and management of glaucoma can effectively reduce its damage to the tissue of the optic nerve and preserve eyesight. In clinical treatment, doctors usually diagnose glaucoma through the size of the intraocular pressure (the normal range is 10–21 mmHg), the vertical diameter ratio of the optic cup (OC) to the optic disc (OD), and the angle between the cornea and the iris [2]. The detection of the optic disc in the retinal fundus images plays an important role in the diagnosis of glaucoma. The OD structure in the fundus images is shown in Figure 1. The shapes of the OD and OC are approximated circular or elliptical and the OC region is inside the OD region. At present, in clinical diagnosis, the extraction of the OD region mainly relies on the doctor's manual marking, which not only takes a long time but also consumes an amount of doctors' energy. In recent years, with the development of computer science, pattern recognition, artificial intelligence, and other disciplines, the computer-aided diagnosis technologies have received more and more concerns. The automatic detection of the OD area in retinal fundus images has become a hot topic.

The article "Fully Convolutional Network and Visual Saliency-Based Automatic Optic Disc Detection in Retinal Fundus Images" was published in 2021. Journal: J Healthc Eng.

The existing OD detection methods can be generally divided into two types: unsupervised learning-based OD detection methods and supervised learning-based OD detection methods. The former OD detection methods based on unsupervised learning can be divided into the following main categories: adaptive threshold-based ones [3,4], superpixel-based ones [5,6], clustering analysis-based ones [7,8], and active contour model-based ones [9–11]. In [3], Issac et al. presented an adaptive threshold method for OD detection. Both means and standard deviations were used to decide the OD region with the interference of the other redundant structures in the red channel images. In [4], Welfer et al. proposed a mathematical morphology-based adaptive method to solve the OD detection problem. Firstly, the intensities were used to detect the OD region roughly, and then the prior shape information of OD was introduced to extract the OD contour accurately. In [5], Cheng et al. developed a superpixel classification-based method for OD detection. Firstly, the fundus images were divided into many superpixels, the features of which were then extracted. According to these features, it is determined whether the superpixel belongs to the OD region or non-OD region. In [6], Rehman et al. firstly performed superpixel segmentation on the fundus images and then extracted the statistical and textural features of each superpixel patch. In the classification stage, four different classifiers were utilized to differentiate between the OD region and background, including Support Vector Machine (SVM), AdaBoost, Random Forest (RF), and RusBoost. In [7], Nija et al. firstly performed Fuzzy C-Means (FCM) clustering algorithm on the morphological preprocessed images, and then the rough detection result was improved by ellipse fitting. In [8], Ma et al. firstly adopted a morphological processing method that considers the characteristics of the vascular structures and gray distribution to extract the region of interest which contains the whole OD area. Secondly, a distance regularized narrow-band level set evolution method was implemented to outline the accurate boundaries of OD. In [9], Gao et al. proposed a novel OD detection model which integrated prior features of OD into the local intensity clustering (LIC) functional energy to eliminate the interference of intensity inhomogeneity, blood vessels, and pathological changes. In addition, this method adopted an improved robust adaptive level set initialization method to deal with the problem associated with the sensitiveness to the initial contour for a better curve evolution result. In [10], Thakur et al. proposed a level set-based adaptive regularization kernel intuitionistic Fuzzy C-Means clustering method to achieve the OD detection. This method firstly used the clustering method to extract the initial contour of the OD area, on the basis of which the level set method is employed to extract the OD area. In [11], Wang et al. considered the geometric structure between the OD and OC and then proposed a two-layer level set method to describe the OD and OC contours. This method can detect the OD and OC boundaries simultaneously. Most of the methods mentioned above have low computational complexity and can be implemented simply. They can achieve the accurate detection of the OD region in fundus images to a certain extent. However, there are still some shortcomings needed to be overcome. These methods can easily suffer from the interference of uneven illumination, low contrast, and blood vessels in fundus images, which results in low accuracy and poor robustness.

The article "Fully Convolutional Network and Visual Saliency-Based Automatic Optic Disc Detection in Retinal Fundus Images" was published in 2021. Journal: J Healthc Eng.

The OD detection methods based on supervised learning can be divided into two major classes: traditional machine learning-based OD detection methods [12–14] and deep learning-based OD detection methods [15–19]. In [12], Niemeijer et al. formulated the detection of OD region in a retinal fundus image as a regression problem. The OD localization was carried out by a trained k-nearest neighbor (KNN) regressor which can measure the distance between the object and a given location. In [13], Acharya et al. proposed a method for OD detection based on texture and local morphological features of fundus images. First, the Leung-Malik filter, Schmid filter, and maximum response filters were used to convolute the fundus image for the extraction of the texture features and the local morphological features. Then these features were utilized to train a desirable classifier to predict outputs. In [14], Perez et al. proposed a novel cascade classifier-based OD detection method. The Haar features extracted from scanning rectangular windows in the fundus images were used for training the cascade classifiers. These traditional machine learning-based OD detection methods are greatly dependent on features extraction and selection. When the selected features cannot accurately distinguish the OD region from the background, the accuracy of the detection methods will be seriously affected. In recent years, deep learning has made great achievements in the fields of image processing and computer vision. The deep learning-based OD detection methods have been widely used due to their excellent feature representation ability. The authors in [20] proposed an elegant fully convolutional network (FCN) architecture named U-net, which can be seen as an outstanding contribution in biomedical image analysis. Most of the follow-up works inherit the core design methodology of U-net. In [15], Sevastopolsky proposed an improved U-net for OD detection. Compared with the original U-net, the modified version designed fewer convolutional layers which can reduce the number of redundant parameters effectively and obtained similar or better detection results. In [16] Edupuganti et al. used an FCN to detect OD regions on full-scale fundus images, and the postprocessing was applied to reduce the false positive noises in the detection results. In [17], Fu et al. proposed a joint multilabel M-net and polar transformation algorithm for OD detection. The performance of OD detection was further improved through a combination of the multiscale pyramid input layers, U-net framework, and multilabel loss function. In [18], Al-Bander et al. proposed an OD detection method that combined Dense Convolutional Network (DenseNet) and FCN to achieve a pixel-level classification result. This network benefited from the dense connection between the current layer and all the previous layers, which achieved feature reuse and mitigated the gradient vanishing problem caused by the increasing of neural network layers. In [19], Yu et al. proposed an improved U-net structure, the core innovation of which was the use of the pretrained ResNet-34 model as the encoding layer. The traditional decoding layer of U-net was still retained to form an integrated OD detection framework. In this way, the introduction of the pretrained ResNet-34 model shortened the training time of the network and thereby further prevented overfitting and improved the robust performance. In [21], Juneja et al. modified U-net architecture by increasing the filter size in the convolution layer, maxpool layer, and upsampling layer, which can achieve higher detection accuracy. In [22], Liu et al. proposed a two-stage method for OD and OC detection. Firstly, the OD is located through a simple convolution neural network. Then the densely connected depthwise separable convolution network (DDSC-Net) was designed to extract the OD and OC according to the localization results. In [23], Jiang et al. proposed a region-based convolutional neural network to detect the OD and OC region. In this network, the disc proposal network and the cup proposal network were constructed to produce bounding box proposals for the OD and OC, respectively. The inscribed ellipses of the corresponding bounding boxes were regarded as the final detection results. These deep learning-based OD detection methods have achieved relatively accurate detection results. However, these models usually require complicated structural design, a large amount of computation, and high hardware requirements. In order to obtain satisfactory results, a large number of data and accurate data annotation from one or more experts are required to be provided to the network, which is difficult to execute.

The article "Fully Convolutional Network and Visual Saliency-Based Automatic Optic Disc Detection in Retinal Fundus Images" was published in 2021. Journal: J Healthc Eng.

In view of the problems above encountered in OD detection, this paper proposes a method of OD detection in fundus images based on FCN and visual saliency. The proposed method shares the advantages of the unsupervised learning-based OD detection methods and the supervised learning-based OD detection methods, which can provide high detection accuracy with low computational complexity. In our method, the optic disc is considered as a salient object and the deep features extracted from a pretrained network without any training are applied to distinguish the OD region from the background. The proposed method mainly contains two stages. First, a morphological reconstruction-based OD localization method [24] is used to locate the OD region in the full-scale fundus images. Then the improved single-layer cellular automata (SCA) model [25] which adopts the deep features extracted from a pretrained FCN [26] for similarity measurement is proposed to extract the accurate optic disc area. The proposed method in this paper is able to overcome the influence of uneven illumination, low contrast, bright lesions, and blood vessel interference in fundus images effectively. A large number of experimental results verify the effectiveness of the proposed method in terms of accuracy and robustness.

The article "Fully Convolutional Network and Visual Saliency-Based Automatic Optic Disc Detection in Retinal Fundus Images" was published in 2021. Journal: J Healthc Eng.

The remainder of this paper is organized as follows. In Section 2, the framework of FCN and SCA is described briefly.  Section 3 provides a detailed description of the proposed OD detection method.  Section 4 presents the experimental results and comparison. Finally, this paper is summarized in Section 5.

## 2. Background

### 2.1. Fully Convolutional Network

In recent years, convolutional neural networks (CNNs) have achieved remarkable results in the field of image processing and computer vision. The main reason is that the CNNs have excellent capabilities in feature representation. They can learn the advanced features with semantic information of the objects [24, 27–29]. CNNs automatically extract features from images by constructing a multilayer convolution structure. The high-level features corresponding to the deeper convolution layer of networks are usually regarded as the abstract expression of object semantic information. As one of the most important CNNs, FCN is an end-to-end semantic segmentation neural network which can accept any size input. Unlike the traditional CNNs for classification tasks, the fully connected layers are totally replaced by the convolutional layers in the FCN. Therefore, all layers in FCN are the convolution layers such that it is called the full convolution network. In the FCN, the deconvolution operations are usually adopted to produce the output with the same size as the input image. The final output assigns each pixel a prediction for the input image to realize the semantic classification at pixel level.  Figure 2 shows the structure of the FCN [26].

FCN is a multilevel neural network, and its different convolutional layers can provide features in multiple scales. In this paper, we use a pretrained FCN [26] to extract the deep features from different layers of the network for the subsequent operation.

### 2.2. Saliency Detection via Single-Layer Cellular Automata

The cellular automata are often seen as a dynamic evolving system with a simple structure and complex self-organizing behavior, which consist of a certain number of cells with discrete states. These cells can evolve according to the specific update rules. During the evolution of each cell, its next state is decided by the current states of itself and its nearest neighbors. Considering that salient objects are spatially coherent, Qin et al. [25] proposed a background-based SCA algorithm, which introduced the cellular automata as an unsupervised propagation mechanism to detect the visual saliency object in the images. Some image features such as color, edge, and texture are often regarded as saliency values to reflect the states of the cells. The similarities in feature space and the distances among cells are utilized to construct the updating strategy. This method can effectively enhance the foreground while suppressing the background by taking into account the intrinsic relationship among cells. Therefore, it can optimize the prior information and update the saliency value to form a dynamic system which can be used to distinguish the target from the background.

The article "Fully Convolutional Network and Visual Saliency-Based Automatic Optic Disc Detection in Retinal Fundus Images" was published in 2021. Journal: J Healthc Eng.

In the SCA-based saliency detection algorithm [25], the Simple Linear Iterative Clustering (SLIC) algorithm [30] is firstly used to segment the image into *N* superpixels, each of which is described by the mean color features and coordinates of pixels. Then the K-means algorithm is adopted to divide the boundary superpixels into *K* clusters as the background seeds according to the features in Lab space. The number of superpixels in cluster *k* can be expressed as *p*^*k*^(*k*=1,2,…, *K*). Consequently, *K* different global color distinction (GCD) maps are constructed according to the *K* superpixel clusters which can be represented as follows:

(1) $$\begin{array}{c} S={\left[s_{k,i}\right]}_{K\times N}, \end{array}$$

where *s*_*k*,*i*_ is the saliency value of superpixel *i* in the *k-*th GCD map and defined by

(2) $$\begin{array}{c} s_{k,i}=\frac{1}{p^{k}}\sum_{j=1}^{p^{k}}\frac{1}{e^{-\left\|c_{i},c_{j}\right\|/2\sigma_{1}^{2}}+\beta }, \end{array}$$

where ‖**c**_*i*_, **c**_*j*_‖ is the Euclidean distance between superpixels *i* and *j* in the Lab color space and *σ*_1_ and *β* are the weight coefficients. In order to integrate the saliency information from each GCD map, the global spatial distance matrix (GSD) is constructed to balance these GCD matrixes, and the GSD matrix is expressed as

(3) $$\begin{array}{c} W={\left[w_{k,i}\right]}_{K\times N}, \end{array}$$

where *w*_*k*,*i*_ represents the spatial distance between superpixel *i* and all boundaries superpixels in the *k*-th cluster and can be expressed as

(4) $$\begin{array}{c} w_{k,i}=\frac{1}{p^{k}}\sum_{j=1}^{p^{k}}e^{-{\left\|r_{i},r_{j}\right\|}_{2}^{2}/2\sigma_{2}^{2}}, \end{array}$$

where **r**_*i*_ and **r**_*j*_ represent the coordinates of superpixels *i* and *j*, respectively, and *σ*_2_ is the weight coefficient.

Integrating the color information *s*_*k*,*i*_ and distance information *w*_*k*,*i*_, the background prior based map *S*^*bg*^=[*S*_*i*_^*bg*^], *i* ∈ [1,…, *N*] is constructed as follows:

(5) $$\begin{array}{c} S_{i}^{bg}=\sum_{k=1}^{K}w_{k,i}\times s_{k,i}, \end{array}$$

where *S*_*i*_^*bg*^ represents the initial saliency value of the *i*-th superpixel at time *t*=0.

Finally, the Euclidean distance ‖**c**_*i*_, **c**_*j*_‖ between superpixels *i* and *j* in the color space is used to construct the impact factor matrix and the coherence matrix. The specified update rules are designed based on these two matrixes to update the saliency value of each superpixel simultaneously. In this way, the salient object detection in the image is realized. In this paper, the optic disc is regarded as a salient object and we improve the SCA-based saliency detection algorithm to extract it.

The article "Fully Convolutional Network and Visual Saliency-Based Automatic Optic Disc Detection in Retinal Fundus Images" was published in 2021. Journal: J Healthc Eng.

## 3. The Proposed Method

The OD is the bright yellowish area which can be regarded as a salient object in the fundus images [24]. In this paper, we introduce the visual saliency detection technique for OD detection and propose a novel OD detection algorithm based on FCN and visual saliency in fundus images. The algorithm flowchart is illustrated in Figure 3. Firstly, the morphological reconstruction-based object detection method is used to locate the OD region roughly and a 400 × 400 red channel image is extracted. Secondly, such an image patch is segmented into many superpixels through the SLIC method. Thirdly, the background prior information and the deep features extracted from the pretrained FCN [26] are to be utilized to represent each superpixel. Finally, both the background prior information and the deep features are integrated into the SCA framework to gain the accurate optic disc detection result.

### 3.1. Optic Disc Region Localization

In the red channel, the OD region usually shows the most contrast against the background. On the contrary, the blood vessels and vascular lesions always appear in low contrast. Therefore, in this paper, we perform the subsequent OD detection operations on the red channel images.  Figure 4 shows an original fundus image and its red channel image.

In this section, we adopt a morphological reconstruction-based object detection method [24] to locate the OD region. Firstly, the Contrast Limited Adaptive Histogram Equalization (CLAHE) algorithm is used to enhance the red channel images, as shown in Figure 5(a). Then, the morphology-based reconstruction method is used to increase the visibility of the OD region, which facilitates the OD region to be obtained. The reconstruction result is shown in Figure 5(b). It is obvious that the OD area appears as a bright structure in the reconstructed image, which means that the OD area contains at least one regional maximum. Therefore, the H-max transform is carried out on the reconstructed image to eliminate all the connected peaks and retrieve a group of OD candidate regions as shown in Figure 5(c). Finally, the maximum coefficient criterion is used to obtain the gravity center of the OD region [31], which is shown in Figure 5(d). In order to detect the OD region more accurately, a square region with a size of 400 × 400 is extracted according to the gravity center of OD, as shown in Figure 5(e). Such an image patch can cover the whole optic disc and the optic disc can be considered as a salient object.

The article "Fully Convolutional Network and Visual Saliency-Based Automatic Optic Disc Detection in Retinal Fundus Images" was published in 2021. Journal: J Healthc Eng.

### 3.2. Visual Saliency-Based OD Detection

#### 3.2.1. Background Priors

For saliency detection, the prior map plays a significant role in locating the salient objects in the image. There are many models proposed to produce such a saliency map. In this paper, we construct a simple prior map which only offers the propagation seeds for improved SCA.

Firstly, we divide the 400 × 400 red channel image into N superpixels by using the SLIC algorithm and compute the average gray value of each superpixel. Then we adopt the Otsu threshold algorithm to obtain a gray threshold to segment the image into background and foreground roughly.

Let *s*_*i*_ ∈ [0,1] be the initial saliency value of superpixel *i* at time *t*=0 which can be decided based on the following assumptions: the superpixels located on the boundary of the image belong to the background and the superpixels whose average gray value is larger than the threshold belong to the object. Therefore, we assign the superpixels on the boundary an initial saliency value close to 0 and the superpixels with larger average gray values an initial saliency value close to 1. For the other superpixels, a uniform initial saliency value is assigned. *s*_*i*_ can be defined by

(6) $$\begin{array}{c} s_{i}=\left\{\begin{array}{cc} 0.9, & s_{i}>\text{threshold,}\\ 0.5, & s_{i}\in \text{others,}\\ 0.01, & s_{i}\in \text{boundaries.} \end{array}\right. \end{array}$$

#### 3.2.2. Extraction of Deep Features in FCN

The traditional SCA model which only adopts the color feature is easily affected by the pathological changes, bright lesions, and complex vascular structures in the fundus image and cannot provide the desirable detection result. It is widely known that the features extracted from the last layer of the CNNs can provide abstract semantic information of objects, which can be used to capture the objects from different complex backgrounds. However, since the spatial resolution of such high-level image features is often low, they cannot represent the spatial detail information effectively. In the CNNs, the low-level features such as edge, color, and texture are usually included in the early layers of the network. Therefore, the combination of these image features extracted from different layers in the network is a benefit for the object description in multiple perspectives. In this paper, we adopt the pretrained FCN (FCN-8s) [26] which is provided by the MatConvNet team to extract deep features from the first pooling layer pool1 and the fifth pooling layer pool5, which are corresponding to the 5th and 31st layers of the network respectively. Some examples of deep feature visualization are shown in Figure 6.

The article "Fully Convolutional Network and Visual Saliency-Based Automatic Optic Disc Detection in Retinal Fundus Images" was published in 2021. Journal: J Healthc Eng.

In the FCN, the deep features in each layer are usually different from each other in resolution because of the operations of subsampling and pooling. Therefore, the features extracted from different layers of network are resized uniformly to the same size of 400 × 400 as the input image by using cropping and nearest neighbor interpolation operations. On this basis, each superpixel can be represented by the means of the deep features corresponding to itself. The similarity measurement between the superpixels *i* and *j* with deep features representation can be defined by

(7) $$\begin{array}{c} g\left(r_{i},r_{j}\right)=\rho \cdot {\left\|df_{i}^{p1}-df_{j}^{p1}\right\|}_{2}+\left(1-\rho \right)\cdot {\left\|df_{i}^{p5}-df_{j}^{p5}\right\|}_{2}, \end{array}$$

where *df*_*i*_^*p*1^ and *df*_*i*_^*p*5^ represent the means of the deep features extracted from pool1 and pool5 corresponding to superpixel *i*, respectively, and *ρ* ∈ [0,1] denotes the weight coefficient to balance the importance between these two features. **r**_**i**_ denotes the feature descriptor of superpixel *i*.

#### 3.2.3. Single-Layer Cellular Automata

In the SCA method, the cells are represented with the superpixels produced by the SLIC approach. The saliency value of each superpixel denotes its current state in the range [0,1]. In this paper, we adopt a more appropriate 2-layer neighborhood for each superpixel. This 2-layer neighborhood of a superpixel includes its adjacent superpixels and the superpixels which share common boundaries with its adjacent superpixels. The next state of each superpixel depends on the current states of itself and its neighborhood superpixels. The saliency values of superpixels are determined by the impact factor matrix and the coherence matrix which are explained as follows.

*(1) The Impact Factor Matrix*. Generally, the next state of a superpixel is greatly influenced by its neighbors which own similar features. The similarity measurement of features between a superpixel and its neighbor is often determined by their distance in the feature space. Therefore, considering an image which is segmented into *n* superpixels, we build an impact factor **F** ∈ **R**^*n*×*n*^ to realize this similarity measurement. We define *f*_*ij*_ as a basic element in **F** ∈ **R**^*n*×*n*^ which represents the impact factor of superpixels *i* to *j* as follows:

(8) $$\begin{array}{c} f_{ij}=\left\{\begin{array}{cc} \exp\left(\frac{-g\left(r_{i},r_{j}\right)}{\sigma_{f}^{2}}\right), & \;j\in \mathrm{NB}\left(i\right),\\ 0, & \;j=i\text{ or others,} \end{array}\right. \end{array}$$

where **r**_*i*_ denotes the feature descriptor of superpixel *i*, *g*(**r**_*i*_, **r**_*j*_) denotes a function which is used to measure the distance between superpixels *i* and *j* in the feature space, *σ*_*f*_ is a weight coefficient to control the strength of *g*(**r**_*i*_, **r**_*j*_), and ***NB***(*i*) represents the set of superpixels in the neighborhood of superpixel *i*. Moreover, a degree matrix **D** is established to regularize the impact factor matrix ***F***.

(9) $$\begin{array}{c} D=\text{diag}\left\{d_{1},d_{2},\ldots ,d_{n}\right\}, \end{array}$$

where *d*_*i*_=∑_*j*_*f*_*ij*_. Finally, the regularized impact factor matrix is formulated as

(10) $$\begin{array}{c} F^{*}=D^{-1}\cdot F. \end{array}$$

*(2) The Coherence Matrix*. The next state of each superpixel is determined by the current state of itself and its neighborhood. Therefore, it is necessary to make a balance between these two factors. When a superpixel is significantly different from its neighborhood in feature space, its next state will mainly depend on itself. On the contrary, when a superpixel is similar to its adjacent neighbors in feature space, its next state will be consistent with them. Based on these analyses, a coherence matrix is constructed to promote the evolution among all superpixels in the following form:

(11) $$\begin{array}{c} C=\text{diag}\left\{c_{1},c_{2},\ldots ,c_{n}\right\}, \end{array}$$

where *c*_*i*_ represents the coherence of each superpixel corresponding to its current state and can be initialized as follows:

(12) $$\begin{array}{c} c_{i}=\frac{1}{\max\left(f_{ij}\right)}. \end{array}$$

Then, the coherence of each superpixel *c*_*i*_ is normalized to be in a range *c*_*i*_ ∈ [*b*, *a*+*b*] with the following form, in which [*b*, *a*+*b*]⊆[0,1]:

(13) $$\begin{array}{c} c_{i}^{*}=a\cdot \frac{c_{i}-\min\left(c_{j}\right)}{\max\left(c_{j}\right)-\min\left(c_{j}\right)}+b, \end{array}$$

where *j*=1,2,…, *n*. Finally, the regularized coherence matrix can be obtained as follows:

(14) $$\begin{array}{c} C^{*}=\text{diag}\left\{c_{1}^{*},c_{2}^{*},\ldots ,c_{n}^{*}\right\}. \end{array}$$

*(3) The Evolution Rule*. All the superpixels will update their states simultaneously according to the evolution rule, which plays a significant role in the final OD detection result. The synchronous evolution rule for all superpixels can be defined as follows:

(15) $$\begin{array}{c} s^{\left(t+1\right)}=C^{*}s^{\left(t\right)}+\left(I-C\right)F^{*}s^{\left(t\right)}, \end{array}$$

where ***I*** represents the *n* × *n* dimensional identity matrix, **F**^*∗*^ and **C**^*∗*^ represent the regularized impact factor matrix and coherence matrix, respectively, and *s*^(*t*)^ ∈ **R**^*n*^ represents the saliency map at time *t*. The initial saliency value **s**^(0)^ of each superpixel can be calculated by (6) corresponding to time *t*=0. Additionally, the evolution rule will not change over time, and the states of all superpixels **s**^(*t*)^ will vary over iterations until convergence.

The article "Fully Convolutional Network and Visual Saliency-Based Automatic Optic Disc Detection in Retinal Fundus Images" was published in 2021. Journal: J Healthc Eng.

There are many bright lesions and complex vascular structures in fundus images, which cause serious interferences for OD detection. The deep features provided by the pretrained FCN [26] have a good performance in distinguishing OD region from different backgrounds. Meanwhile, the SCA method makes use of the correlation adequately among the adjacent regions to enhance the saliency of the regions with similar features. Therefore, the proposed method can overcome these interferences and yield desirable detection results.

## 4. Experimental Results and Analysis

In order to verify the effectiveness of the proposed method, the proposed method is applied to carry out OD detection and compared with some existing OD detection methods including the improved circular Hough transform and superpixel segmentation method based on Hough peak selection (SLIC-Hough) [32], local intensity clustering model based on the fusion of multiple features (LICE) (Gao et al.) [9], and the dense U-net method that combines DenseNet and full convolutional neural network [18] which is trained on HP Z440 workstation for 120 epoch with 15 hours used.

The compared experiments are performed on two public retinal fundus image datasets: DRISHTI-GS dataset [32] and RIM-ONE r3 dataset [33]. The DRISHTI-GS dataset is provided by Aravind Eye Hospital, Madurai, India, which can be used to verify the performance of computer-aided algorithms. This dataset contains 101 color retinal fundus images with a resolution of 2896 × 1944 and a field of view of 30° centered at OD. The ground truth of each image is annotated manually by four experts with many years of clinical experience. The RIM-ONE r3 dataset collects 169 color retinal fundus images, the ground truth of which is created by five experienced ophthalmic experts. In order to evaluate the performance of the proposed OD detection method in qualitative and quantitative, the Dice coefficient, Jaccard coefficient, recall coefficient, and accuracy evaluation metrics are adopted to measure the detection results. The values of evaluation indexes above all range from 0 to 1, and the larger these evaluation indexes are, the better the OD detection results are. In the following, the true positive (TP), false positive (FP), true negative (TN), and false negative (FN) are used to explain the evaluation indicators above.

The article "Fully Convolutional Network and Visual Saliency-Based Automatic Optic Disc Detection in Retinal Fundus Images" was published in 2021. Journal: J Healthc Eng.

The Dice coefficient is defined by

(16) $$\begin{array}{c} \text{Dice}=\frac{2\times TP}{2\times TP+FP+FN}, \end{array}$$

where the Dice coefficient represents the ratio of the overlap region between the detection result and the ground truth to the total region.

The Jaccard coefficient that measures the similarity between the detection result and the ground truth is defined by

(17) $$\begin{array}{c} \text{Jac}=\frac{\text{TP}}{\text{TP}+\text{FP}+\text{FN}}. \end{array}$$

The recall coefficient that represents the ability of the method to detect the object is defined by

(18) $$\begin{array}{c} \text{Rec}=\frac{\text{TP}}{\text{TP}+\text{FN}}. \end{array}$$

The accuracy that reflects the ratio of the correctly detected regions to the whole result is defined by

(19) $$\begin{array}{c} \text{Acc}=\frac{\text{TP}+\text{TN}}{\text{TP}+\text{TN}+\text{FP}+\text{FN}}. \end{array}$$

The parameter setting in this experiment is as follows: *n*=200, *ρ*=0.35, 1/*σ*_*f*_^2^=23, *a*=0.9, and *b*=0. All of these parameters are decided according to a large number of experiments. And the experiments are carried on a computer with i7-4710MQ CPU at 2.50 GHz, 64 GB of RAM, and Matlab2019a.

Figure 7 shows the comparisons among these four methods to detect the OD region on retinal fundus images with complex vascular structures.  Figure 7(a) shows the original fundus images.  Figure 7(b) shows the ground truth. Figures 7(c)–7(f) show the OD detection results by the proposed method, the SLIC-Hough method, the LICE method, and the modified U-net method, respectively. From these experimental results, it can be seen that the SLIC-Hough method is severely interfered with by these complex vascular structures. Though it always tends to extract the OD region which approximates an ellipse shape, the fitting ellipses deviate greatly from the ground truth. The LICE method suffers from the influence of blood vessels seriously, which results in inaccurate boundaries of OD regions. The modified U-net method is also affected by the blood vessels. When the blood vessels are densely distributed, it cannot produce desirable detection results. Compared with these three methods, the proposed method is able to overcome the interference of blood vessels effectively and obtain the best OD detection result.

Figure 8 shows the detection results of four methods on some fundus images with weak OD boundaries and low contrast between the OD regions and the background. Figure 8 displays the OD detection results in some fundus images with many lesion areas and irregular OD shapes.  Figure 8(a) shows the original fundus images.  Figure 8(b) shows the ground truth. Figures 8(c)–8(f) show the OD detection results by the proposed method, the SLIC-Hough method, the LICE method, and the modified U-net method, respectively. It is obvious that the SLIC-Hough method cannot capture the boundaries of the OD correctly, which causes that the fitting ellipse deviates greatly from the ground truth. The LICE method is sensitive to weak edges and yields the worst OD detection results. The modified U-net method always tends to detect the brightest part in the OD region which leads to inaccurate OD detection results. Instead, the proposed method that benefits from the deep features extracted from the pretrained FCN [26] is less affected by the blur OD boundaries and the low contrast and obtains the desirable OD detection results.

The article "Fully Convolutional Network and Visual Saliency-Based Automatic Optic Disc Detection in Retinal Fundus Images" was published in 2021. Journal: J Healthc Eng.

Figure 9 displays the OD detection results on some fundus images with many lesion areas and irregular OD shapes.  Figure 9(a) shows the original fundus images.  Figure 9(b) shows the ground truth. Figures 9(c)–9(f) show the OD detection results by the proposed method, the SLIC-Hough method, the LICE method, and the modified U-net method, respectively. By the analysis of the experimental results, we evaluate the performance of these methods as follows. The SLIC-Hough method always considers the OD region as an ellipse shape, even when the shape of the OD is seriously irregular due to the influence of the ocular diseases. Additionally, the lesions around the OD area are also regarded as the OD region. The LICE method suffers from the interference of the lesions severely. When the intensities between the OD region and lesions are close to each other, the method is not able to distinguish them correctly. The modified U-net method is seriously affected by the lesion in the fundus images, and some lesions cannot be distinguished from the OD region. Compared with the methods mentioned above, the proposed method can overcome the influence of lesion interference to a certain extent and extract the OD boundaries more accurately.

In order to further verify the performance of these OD detection methods, we compare the proposed method with the other approaches according to the numerical indices mentioned above for quantitative analysis.  Table 1 shows the experimental results obtained by four different methods on the DRISHTI-GS and RIM-ONE r3 datasets. By observing the numerical data in the table, it can be seen that the proposed method is superior to other methods in terms of the Dice, Jaccard, and recall coefficients. As for the accuracy evaluation indexes, our method and the supervised deep learning-based modified U-net method have achieved similar results and are higher than the other approaches.

The article "Fully Convolutional Network and Visual Saliency-Based Automatic Optic Disc Detection in Retinal Fundus Images" was published in 2021. Journal: J Healthc Eng.

According to the results and analysis of the above qualitative experiments, it can be seen that the algorithm in this paper can effectively overcome the interference of multiple tissues such as uneven grayscale, low brightness, blood vessels, and lesions in fundus images and achieve accurate detection of the OD area. These experimental results demonstrate its effectiveness and robustness.

## 5. Conclusions

In this paper, we present a novel unsupervised learning approach for OD detection based on FCN and visual saliency detection in retinal fundus images. We focus on the accurate extraction of the OD region with the interference of vascular structures, lesion areas, and intensity inhomogeneity. The morphological reconstruction-based-based object detection method is utilized first to achieve the rough localization of the OD region. On this basis, the improved SCA model which incorporates the deep features extracted from a pretrained FCN [26] into the original framework is proposed to extract the accurate optic disc area. Our proposed OD detection method is evaluated on the DRISHTI-GS dataset and the RIM-ONE r3 dataset. The experimental results and quantitative analysis demonstrate that the proposed method is able to detect the OD regions precisely and yields superior performance compared with some existing methods.

## Figures and Tables

**Figure 1:** Optic disc region in retina fundus image.

**Figure 2:** The structure of the FCN.

**Figure 3:** The flowchart of the proposed method.

**Figure 4:** (a) The original fundus image and (b) its red channel image.

**Figure 5:** The extraction of OD region. (a) The enhanced red channel map; (b) morphological reconstruction map; (c) binary map of candidate regions; (d) the gravity center of OD region; (e) the cropped OD region.

**Figure 6:** Some examples of deep feature visualization.

**Figure 7:** The OD detection results of four methods on retinal fundus images with complex vascular structures. (a) The original fundus images; (b) the ground truth; (c) results of ours; (d) results of SLIC-Hough method; (e) results of LICE method; (f) results of modified U-net method.

**Figure 8:** The OD detection results of four methods on retinal fundus images with weak boundaries. (a) The original fundus images; (b) the ground truth; (c) results of ours; (d) results of SLIC-Hough method; (e) results of LICE method; (f) results of modified U-net method.

**Figure 9:** The OD detection results of three methods on retinal fundus images with lesions and irregular OD shapes. (a) The original fundus images; (b) the ground truth; (c) results of ours; (d) results of SLIC-Hough method; (e) results of LICE method; (f) results of modified U-net method.

The article "Fully Convolutional Network and Visual Saliency-Based Automatic Optic Disc Detection in Retinal Fundus Images" was published in 2021. Journal: J Healthc Eng.

**Table 1:** Comparison of the evaluation indexes with different methods.

Methods	Dataset	Dice	Jaccard	Recall	Accuracy
SLIC-Hough	DRISHTI-GS	0.866 3	0.846 7	0.953 4	0.992 2
	RIM-ONE r3	—	—	—	—
LICE	DRISHTI-GS	0.920 0	0.854 1	0.935 2	0.967 9
	RIM-ONE r3	0.905 6	0.810 7	0.896 4	0.924 1
Modified U-net	DRISHTI-GS	0.949 0	0.904 2	0.926 8	0.996 9
	RIM-ONE r3	0.903 6	0.8289	0.8737	0.9922
Our method	DRISHTI-GS	0.965 8	0.934 1	0.964 8	0.996 7
	RIM-ONE r3	0.918 2	0.877 5	0.904 8	0.993 2

## Data Availability

The data used to support the findings of this study are available from the corresponding author upon request.
